The article "Expression and Related Mechanisms of miR-100 and TRIB2 in COPD Patients" was retracted in 2023. Reasons: signs of a paper mill; suspected computer-generated content; unreliable results or conclusions; concerns about the data.

# Expression and Related Mechanisms of miR-100 and TRIB2 in COPD Patients

**DOI:** 10.1155/2022/6556208

**Published:** 2022-04-21

**Authors:** Zhitao Mai, Ya Mi, Mingming Jiang, Shanzhi Wan, Qingguo Di

**Affiliations:** ^1^Department of Respiratory and Critical Care Medicine, Cangzhou Central Hospital, Cangzhou 061001, Hebei, China; ^2^Hemodialysis Room, Cangzhou Central Hospital, Cangzhou 061001, Hebei, China

## Abstract

**Background:**

Chronic obstructive pulmonary disease (COPD) is one of the most common chronic respiratory diseases in the world. COPD is a general term for a class of lung diseases, including emphysema, chronic bronchitis, and refractory asthma. It is characterized by irreversible airflow obstruction and chronic tracheal inflammation.

**Objective:**

This study aimed to investigate the expression and related mechanisms of miR-100 and TRIB2 in patients with COPD.

**Methods:**

We collected the serum of patients admitted to our hospital and healthy volunteers undergoing physical examination at the same time, pulmonary fibroblasts were purchased for the experiments, miR-100 was overexpressed, and TRIB2 expression was inhibited in cells. The miR-100 and TRIB2 expression levels in serum and cells were detected by qRT-PCR and Western blot, cell proliferation and apoptosis were detected by CCK-8 and flow cytometry, and the relationship between miR-100 and TRIB2 was explored by the dual-luciferase report.

**Results:**

The miR-100 expression in the serum of the COPD group was expressed normally, while the TRIB2 expression was expressed abnormally (*p* < 0.05). The AUC of serum miR-146a and TRIB2 for COPD diagnosis were 0.965 and 0.954, respectively. Overexpressing miR-100 and inhibiting the TRIB2 expression could decrease cell proliferation and increase apoptosis rate. According to the dual-luciferase report, miR-100 and TRIB2 had a targeted regulatory relationship. Rescue experiments showed that overexpressing TRIB2 could reverse the changes of cell proliferation and apoptosis caused by overexpression of miR-100.

**Conclusion:**

miR-100 and TRIB2 were expressed abnormally in serum of COPD patients, and miR-100 could inhibit proliferation of pulmonary fibroblasts and promote their apoptosis.

## 1. Introduction

Chronic obstructive pulmonary disease (COPD) is one of the most common chronic respiratory diseases in the world. COPD is a general term for a class of lung diseases, including emphysema, chronic bronchitis, and refractory asthma. Its symptoms are shortness of breath, cough, and sputum production. It is characterized by irreversible airflow obstruction and chronic tracheal inflammation. According to statistics, about 3 million people worldwide die of COPD every year [1, 2]. With the passage of time, patients will face worsening acute symptoms and gradual decline of lung function, resulting in more difficult daily activities of patients and serious decline in life therapy. As to the treatment of COPD, drug therapy is mainly adopted clinically, including short-term or long-term use of *β*-2 agonists and anticholinergic drugs, corticosteroids, and methylxanthine. However, these drugs cannot slow down lung function and improve survival rates [3]. Although COPD involves many aspects, including oxidative stress, the imbalance between proteolytic and anti-proteolytic activities, immunity and inflammation, apoptosis, and repair and destruction of airway and lung, its exact pathogenesis is still unclear [4]. Given the harm of COPD to people and the current difficulties in treatment, it is necessary to clarify the relevant mechanism of COPD pathogenesis. Only the pathogenesis of COPD needs to be clarified in order to improve the treatment level.

The article "Expression and Related Mechanisms of miR-100 and TRIB2 in COPD Patients" was retracted in 2023. Reasons: signs of a paper mill; suspected computer-generated content; unreliable results or conclusions; concerns about the data.

MicroRNA (miRNA, miR) is a single-stranded non-coding RNA composed of about 23 nucleotides, which can participate in a variety of cell biological processes, such as proliferation and apoptosis [5, 6]. It is estimated that miR can regulate one-third of human genes and affect their functions and genetic pathways [7]. The miR-99 family was made up of miR-100 and miR-99a\b [8]. Many studies have found that miR-100 participates in the occurrence and development of diseases. For example, some research results showed that miR-100 could act as a tumor suppressor gene in esophageal cancer and gastric cancer through targeted regulation of CXCR7 [9, 10]. Other studies revealed that miR-100 could inhibit the migration and invasion of nasopharyngeal carcinoma cells by targeting IGF1R [11]. In recent years, some studies have found that miR-100 is expressed low in serum of COPD patients [12], but they have not explored the relationship between miR-100 and COPD. We have discovered a targeted binding site between Tribbles homolog 2 (TRIB2) and miR-100 through online biological prediction software. TRIB2 belongs to one of the members of the Tribbles family, and the members of this family play the part of scaffold protein in the signal transmission process [13]. TRIB2 is considered to be an oncogene and participates in the biological functions of disease cells. For instance, there were research results showing that TRIB2 was highly expressed in small cell lung cancer, and its overexpression could promote cisplatin resistance by reducing the level of enhancer-binding protein *α* in small cell lung cancer cells [14]. Other research results indicated that TRIB2 was also highly expressed in colon cancer, and the high expression of TRIB2 showed a poor prognosis of colon cancer patients. However, we did not know which way miR-100 affected the apoptosis and proliferation of pulmonary fibroblasts. They also demonstrated that TRIB2 could accelerate cell growth, cycle progression, and prevent cell senescence by blocking AP4/p21 signal conduction [15].

The article "Expression and Related Mechanisms of miR-100 and TRIB2 in COPD Patients" was retracted in 2023. Reasons: signs of a paper mill; suspected computer-generated content; unreliable results or conclusions; concerns about the data.

Therefore, we proposed the conjecture of “whether miR-100 can inhibit COPD progression through targeted TRIB2.” In order to confirm this, we carried out the following research. We used qRT-PCR and Western blot to explore the miR-100 and TRIB2 expression levels in serum and cells. We also used CCK-8 and flow cytometry to explore cell proliferation and apoptosis. The relationship between miR-100 and TRIB2 was explored by the dual-luciferase report.

## 2. Materials and Methods

### 2.1. General Information

The subjects of this study were 88 COPD patients (COPD group) treated in our hospital from March 2018 to February 2019. The inclusion criteria were as follows: those who complied with COPD diagnostic criteria [16], those between 50 and 70 years old, those with complete clinical data, and those who quit smoking for more than 10 years. Exclusion criteria were as follows: severe functional loss of respiratory diseases, tumors, liver, kidney and other important organs except for COPD; those with communication difficulties; and those with poor compliance. Another 60 volunteers who underwent physical examination in our hospital during the same period were recruited as the normal group. The inclusion criteria included those who had no previous chronic respiratory disease, smoking history or major diseases, and had no difference between the patients and general clinical data such as age, gender, height and weight, and place of residence. Patients in both groups signed informed consent, and this study was also approved by the Ethics Committee.

### 2.2. Collection of Serum Samples

A total of 5 ml of fasting venous blood was drawn from patients in the two groups in the early morning into a centrifuge tube, and then, it was centrifuged 15 min at 3000 r/min, and finally, the supernatant was taken and placed in a −80°C refrigerator to be tested.

### 2.3. Cell Source and Treatment

Peripheral airway fibrosis is considered to be an important cause of COPD, and its main process is the proliferation of pulmonary fibroblasts [17, 18]. Therefore, MRC-5, a lung fibroblast from ATCC, was selected as the cell object of the cell experiment. The purchased MRC-5 was transferred into a DMEM low-glucose medium (Gibco, USA) containing a penicillin-streptomycin double antibody and 10% FBS, and it was cultured in 37°C, 5% CO_2_. Targeted elevation miR-100 (miR-100-mimics), miR negative control (miR-NC), targeted inhibition TRIB2 RNA (si-TRIB2), and negative control RNA (Si-NC) were transfected into MRC-5 by a Lipofectamine™ 2000 kit, the operation steps were strictly carried out according to the kit instructions, and then it was cultured for one day.

The article "Expression and Related Mechanisms of miR-100 and TRIB2 in COPD Patients" was retracted in 2023. Reasons: signs of a paper mill; suspected computer-generated content; unreliable results or conclusions; concerns about the data.

### 2.4. Detection Methods

#### 2.4.1. qRT-PCR

The total RNA in cells and serum was extracted according to the instructions of the TRIzol extraction kit (Chundu Biotechnology Co., Ltd., Wuhan, China), the concentration and purity of total RNA were detected by an ultraviolet-visible spectrophotometer (Scientific Equipment Co., Ltd., Hangzhou, China) and agarose gel electrophoresis, and then RNA was reverse transcribed into cRNA in the light of the instructions of a reverse transcription kit (Tiangen Biochemical Technology Co., Ltd., Beijing, China, one-step method). Soon afterward, the reaction system of PCR amplification was as follows: 2 × Talent qPCR PreMix 10 *μ*l, upstream and downstream primers each 1.25 *μ*l, cDNA 100 ng, water added to 20 *μ*l. Reaction conditions were as follows: pre-denaturation at 95°C for 3 min, denaturation at 95°C for 5 s, and annealing extension at 60°C for 15 s, with 40 cycles. The data were analyzed using 2^−△△CT^.

#### 2.4.2. Western Blot (WB)

Protein was extracted from cells of each group using the RIPA lysis method, and its concentration was detected with a BCA kit (Thermo Scientific™) and adjusted to 4 *μ*g/*μ*L. The proteins were separated by 12% SDS-PAGE electrophoresis and then transferred to a PVDF membrane. The membrane was stained with Ponceau S working solution, immersed 5 min in PBS and then washed, blocked 2 h with 5% skimmed milk powder, added with TRIB2 (1 : 1000) and *β*-catenin (1 : 1000) primary antibodies (Abcam, USA), and incubated overnight at 4°C. After washing the membrane, a horseradish peroxidase-labeled goat anti-rabbit II antibody (R&D, USA) (1 : 5000) was added, and then it was incubated for 1 h at 37°C, rinsed 3 times with PBS for 5 min each time. The protein was developed using the enhanced chemiluminescence (ECL) reagent, the protein bands were scanned, and the gray values were analyzed by a Gel-Pro analyzer. The relative expression level of each protein = the gray value of the target protein band/the gray value of the *β*-Actin protein band.

#### 2.4.3. Cell Proliferation Test (CCK-8)

The transfected cells were adjusted to 4*∗*10^4^ and inoculated on 96-well plates. The CCK-8 kit (Beyotime Biotechnology, Shanghai, China) was used for detection. After the cells were transfected for 24 h, they were collected, adjusted to 4*∗*10^6^, inoculated on 96-well plates, and then were cultured for 24, 48, 72, and 96 h. After that, 10 *μ*L of CCK8 solution and 90 *μ*L of DMEM were added to each well, cultured 2 h at 37°C, and then the OD value of cells was measured at 490 nm absorbance by an enzyme labeling instrument.

The article "Expression and Related Mechanisms of miR-100 and TRIB2 in COPD Patients" was retracted in 2023. Reasons: signs of a paper mill; suspected computer-generated content; unreliable results or conclusions; concerns about the data.

#### 2.4.4. Apoptosis Detection (Flow Cytometry)

The transfected cells were digested with 0.25% trypsin and washed with pre-cooled 0.01 mol/L PBS. After the cells were centrifuged, the supernatant was discarded, a 100 *μ*L binding buffer was used to suspend them, and then they were transferred to flow detection tubes. AnnexinV-FITC and PI (Yuduo Biotechnology Co., Ltd., Shanghai, China) were sequentially added to each tube, the cells were reacted 10 min in a dark room, and flow cytometry (BD, USA, FACS Canto II) was used for detection. Each sample was repeatedly detected 3 times.

#### 2.4.5. Detection of Target Genes

TargetScan7.2 biological prediction website was used to predict the target gene downstream of miR-100. TRIB2-3'UTR wild type (Wt) and TRIB2-3'UTR mutant (Mut) were transfected into MRC-5 based on the Lipofectamine™ 2000 kit instructions, and luciferase activity was detected according to the instructions of a dual-luciferase report gene detection kit (Solarbio, Beijing, China).

### 2.5. Statistical Analysis

SPSS 21.0 (IBM Corp, Armonk, NY, USA) was used to analyze the data collected in this paper, and GraphPad 7 software package was used to draw pictures. The comparison between the mean values of the two groups was conducted by *t*-test. One-way analysis of variance was used for the comparison between mean values of more than two groups, and Dunnett-t test was used for the later two comparisons. A *p*-value lower than 0.05 was considered statistically significant.

## 3. Results

### 3.1. Expression and Diagnostic Value of miR-100 and TRIB2 in COPD Patients

Based on the gene expression of miR-100 and TRIB2 in serum, the miR-100 expression in serum of the COPD group was lower than that of normal group, while the TRIB2 expression was just the opposite (*p* < 0.05). Taking the median values of miR-100 and TRIB2 expression in COPD group as critical points, we analyzed the relationship between the two expression levels and the pulmonary function of patients. The results showed that the lower miR-100 and the higher TRIB2 were tied to the poor lung function (Figure 1).

### 3.2. Effect of miR-100 on Proliferation and Apoptosis of MRC-5 Cells

In order to explore the role of miR-100 in COPD, the proliferation and apoptosis of MRC-5 cells were observed after they were transfected with miR-100-mics and miR-NC. The results showed that the miR-100 expression in the transfected miR-100-mics cells increased, and the cell proliferation was inhibited, while the apoptosis rate increased (Figure 2).

The article "Expression and Related Mechanisms of miR-100 and TRIB2 in COPD Patients" was retracted in 2023. Reasons: signs of a paper mill; suspected computer-generated content; unreliable results or conclusions; concerns about the data.

### 3.3. Effect of TRIB2 on Proliferation and Apoptosis of COPD Cells

In order to explore the role of TRIB2 in COPD, this paper treated MRC-5 cells with TRIB2 inhibition, and we observed the changes in cell proliferation and apoptosis after treatment. The results showed that after transfection, the TRIB2 expression decreased, the proliferation of cells was inhibited, and the apoptosis rate increased (Figure 3).

### 3.4. Dual-Luciferase Report

After predicting miR-100 downstream target genes through the TargetScan website, we found that miR-100 and TRIB2 had targeted binding sites. According to the dual-luciferase activity detection results, we found that after miR-100 was overexpressed, the TRIB2 3'UTR Wt luciferase activity was inhibited (*p* < 0.05), but it had no effect on the TRIB2 3'UTR Mut luciferase activity (*p* > 0.05). WB detection results showed that the TRIB2 expression in miR-100-mimics transfected cells was lower than that in miR-NC transfected cells (*p* < 0.05) (Figure 4).

### 3.5. Effect of Overexpression of miR-100 and TRIB2 on Proliferation and Apoptosis of MRC-5 Cells

After detecting of miR-NC, we transfected miR-100-mimics + sh-TRIB2 and miR-100-mimics into MRC-5 cells, respectively, and discovered that there was no difference between the proliferation and apoptosis of the transfected miR-100-mimics + sh-TRIB2 cells and those of the transfected miR-NC cells, but the proliferation increased and the apoptosis rate decreased compared with those of the transfected miR-100-mimics cells (Figure 5).

## 4. Discussion

COPD is one of the most common chronic respiratory diseases in the world. COPD is a general term for a class of lung diseases, including emphysema, chronic bronchitis, and refractory asthma. Its symptoms are shortness of breath, cough and sputum production [19, 20]. Although COPD is a serious and increasing global burden disease, it is incurable at present. With the passage of time, patients will face worsening acute symptoms and gradual decline of lung function, resulting in more difficult daily activities of patients and serious decline in life therapy [21, 22]. Therefore, only the pathogenesis of COPD needs to be clarified in order to improve the treatment level.

The miR expression imbalance exists in patients with various diseases and participates in the occurrence and development of various diseases including COPD [22–25]. As a member of miR, miR-100 is found to be low expressed in serum of COPD patients in previous studies [12]. This study once again proved that miR-100 was expressed low in serum of COPD patients, and its low expression was related to poor lung function, which indicated that miR-100 might participate in the progression of COPD. Next, we conducted cell experiments. We used CCK-8 and flow cytometry to explore cell proliferation and apoptosis. We also adapted qRT-PCR and Western blot to explore the miR-100 and TRIB2 expression levels in serum and cells. The relationship between miR-100 and TRIB2 was detected by the dual-luciferase report. The experimental results showed that overexpressed miR-100 could reduce the proliferation of pulmonary fibroblasts and increase their apoptosis rate, which implied that miR-100 was expected to become one of the targets for treating COPD. However, we did not know the mechanism by which miR-100 affected the apoptosis and proliferation of pulmonary fibroblasts.

The article "Expression and Related Mechanisms of miR-100 and TRIB2 in COPD Patients" was retracted in 2023. Reasons: signs of a paper mill; suspected computer-generated content; unreliable results or conclusions; concerns about the data.

We found that TRIB2 was predicted as a potential target of miR-100 by online biological prediction software. TRIB2 was identified as a serine/threonine kinase of an oncogene [26]. It could be targeted and regulated by various miRs, thus affecting the progression of diseases. For example, research results showed that miR-99 in cervical cancer could inhibit cell proliferation and promote apoptosis through targeted TRIB2. Other showed that miR-511 and miR-1297 inhibited the proliferation of human lung adenocarcinoma cells by targeting TRIB2. Previous studies have not revealed which way miR-100 affected the apoptosis and proliferation of pulmonary fibroblasts. These studies revealed that miR/TRIB2 axis played a key role in diseases. In our study, we innovatively found that the high expression of TRIB2 was tied to poor pulmonary function and TRIB2 was highly expressed in serum of patients with COPD. Subsequently, through cell experiments, we found that inhibiting the TRIB2 expression in pulmonary fibroblasts could reduce the cell proliferation and promote the apoptosis rate, which suggested that TRIB2 was also one of the therapeutic targets for COPD. Then, we found that the proliferation and apoptosis of miR-100-mimics + sh-TRIB2 cells were not different from those of miR-NC cells, while the proliferation increased and the apoptosis rate decreased compared with miR-100-mimics cells. We also confirmed the relationship between TRIB2 and miR-100. We found that after miR-100 was overexpressed, the activity of TRIB2 3'UT Wt luciferase reduced, but the activity of TRIB2 3'UTR Mut luciferase did not change. Besides, the TRIB2 expression in miR-100-mimics transfected cells was lower than that in miR-NC transfected cells. The abovementioned research results preliminarily prove that miR-100 could promote COPD apoptosis by targeting TRIB2.

The article "Expression and Related Mechanisms of miR-100 and TRIB2 in COPD Patients" was retracted in 2023. Reasons: signs of a paper mill; suspected computer-generated content; unreliable results or conclusions; concerns about the data.

## 5. Conclusion

This research confirmed that miR-100 and TRIB2 had a targeted regulatory relationship. Rescue experiments showed that overexpressing TRIB2 could reverse the changes of cell proliferation and apoptosis caused by overexpression of miR-100. This study preliminarily proved that miR-100 and TRIB2 were abnormally expressed in serum of COPD patients, and miR-100 could inhibit proliferation of pulmonary fibroblasts and promote their apoptosis. This was expected to become a potential indicator target clinically.

However, this study still has limitations. For example, we did not understand the relationship between the miR-100 and TRIB2 expression levels and the survival of patients due to the short time and the small number of collected samples. Besides, we did not conduct animal experiments, so we did not know the impact of miR-100 and TRIB2 on COPD pathology. Our future research direction is to solve the limitations of this study. First, we will conduct animal experiments.

## Figures and Tables

**Figure 1:** Expression of miR-100 and TRIB2 in COPD patients. (a) miR-100 expression in serum of COPD group is lower than that of normal group. (b) TRIB2 expression in serum of COPD group is higher than that of normal group. (c) Lower miR-100 is associated with poor lung function. (d) High TRIB2 is associated with poor lung function. ^*∗*^*p* < 0.05; FEV1 (%): the percentage of forced expiratory volume in one second shared by forced vital capacity.

**Figure 2:** Effect of miR-100 on proliferation and apoptosis of MRC-5 cells. (a) miR-100 expression in transfected miR-100-mimics cells increases. (b) Cell proliferation of transfected miR-100-mimics is inhibited. (c) Apoptosis rate of miR-100-mimics transfected cells increases. ^*∗*^*p* < 0.05.

**Figure 3:** Effect of TRIB2 on proliferation and apoptosis of MRC-5 cells. (a) TRIB2 expression in transfected si-TRIB2 cells decreases. (b) Proliferation of cells transfected with si-TRIB2 is inhibited. (c) Apoptosis rate of si-TRIB2 transfected cells increases. ^*∗*^*p* < 0.05.

**Figure 4:** Dual-luciferase report. (a) Through the TargetScan website, we predict that miR-100 and TRIB2 have targeted binding sites. (b) After miR-100 is overexpressed, TRIB2 3'UTR Wt luciferase activity is inhibited, but it has no effect on TRIB2 3'UTR Mut luciferase activity. (c) TRIB2 expression in miR-100-mimics transfected cells is lower than that in miR-NC transfected cells. ^*∗*^*p* < 0.05.

**Figure 5:** Comparison of miR-100-mimics + sh-TRIB2, miR-100-mimics, and miR-NC. (a) There is no difference between proliferation of cells transfected with miR-100-mimics + sh-TRIB2 and that of miR-NC cells, while the proliferation of cells transfected with miR-100-mimics increases. (b) There is no difference between apoptosis of miR-100-mimics + sh-TRIB2 cells and that of miR-NC cells, while the apoptosis rate of miR-100-mimics cells is lower than that of miR-100-mimics cells. ^*∗*^*p* < 0.05.

The article "Expression and Related Mechanisms of miR-100 and TRIB2 in COPD Patients" was retracted in 2023. Reasons: signs of a paper mill; suspected computer-generated content; unreliable results or conclusions; concerns about the data.

## Data Availability

The datasets used and/or analyzed during the current study are available from the corresponding author on reasonable request.
